# A Performance Comparison of Classification Algorithms for Rose Plants

**DOI:** 10.1155/2022/1842547

**Published:** 2022-08-16

**Authors:** Muzamil Malik, Waqar Aslam, Emad Abouel Nasr, Zahid Aslam, Seifedine Kadry

**Affiliations:** ^1^Department of Computer Science & Information Technology, The Islamia University of Bahawalpur, Bahawalpur, Pakistan; ^2^Industrial Engineering Department, College of Engineering, King Saud University, Riyadh 11421, Saudi Arabia; ^3^Department of Applied Data Science, Noroff University College, Kristiansand, Norway

## Abstract

One of the key roles of Botanists is to be able to recognize flowers. This role has become highly challenging given that the number of discovered flower types are nearing half a million. To support Botanists, Information Technology offers promising solutions. Specifically, machine learning techniques are intrinsically appealing due to being precise enough as required. To this aim, two observations on flower leaves are relevant and leverage flower identification: one, flower plants exhibit unique features in their leaves thus allow distinction of their co-located flowers; two, leaves have a much longer life than flowers thus preserve identity properties longer. This paper proposes the use of machine learning-based identification of rose types by leveraging the features from their leaves. For this purpose, the performance of Naive Bayes, Generalized Linear Model, Multilayer Perceptron, Decision Tree, Random Forest, Gradient Boosted Trees, and Support Vector Machine has been analyzed. This study optimizes the RF model by investigating and tuning its various parameters such as the number of trees, the depth of trees, and splitting criteria. The best results are achieved with gain ratio because it takes more distinct values to avoid the problems associated with Information Gain. Optimizing the number of trees and the depth of trees of RF yield better accuracy than other models. Extensive experiments are performed to analyze the results of ensemble algorithms by using the voting method for each instance. Results suggest that the performance of ensemble classifiers is superior to that of individual models.

## 1. Introduction

Pakistan has an agriculture-based economy in which the horticulture profession is common. For agriculture implants, most traditional resources are used and the population is massively growing due to which national production requirements are hardly met. The cost-benefit ratio in the agriculture industry is suboptimal and requires the adoption of new technologies and automated processes. To this end, one interesting area of automation is image processing for effective usage in horticulture. Machine learning in image processing has met great success to solve real-world problems such as detection and classification of cancerous tissues, face recognition, crop/plant classification, and image-based searching [1].

Plant classification has been a very important research area for many decades. So far about 250,000 kinds of flowering plants have been identified and classified [2]. Researchers have been trying to make the classification of fruit, vegetable, and flowering plants an easy process with lesser manual involvement. Amongst flowering plants, rose plants have universal appeal due to their matchless beauty. They have economic value due to demand around the globe as being used to prepare medicines, cosmetics, perfumes, oils, etc. [3]. The Netherlands is home to the largest rose farms in the world [4]. It is increasingly becoming relevant and significant to keep track of not only existing rose species but also to identify new ones.

Rose plants vary in their morphological characteristics, which may affect their leaves, flowers or even the entire plants [5]. Rose leaves contain key knowledge and survive longer than the roses. Identifying rose plants or in general flowering plants through their leaves is a troublesome task for plant scientists if done manually. It requires appropriate training, time, and manpower to perform this task, especially if done at a larger scale. Given that roses have about 150 species that vary in colours, sizes, and fragrance, their manual identification is still tedious and time-consuming. There is a need for an efficient approach, adopting which this task can be performed on large scale using the available automation technologies. Thus, the main objective of this work is to identify rose types automatically. With the high availability of smart mobile phones, the idea is to develop an expert application that can classify roses, thus effectively eliminating the involvement of plant scientists. This application can use the built-in phone camera to capture rose leave images for roses classification [5]. To this end, our preliminary work is based on the k-nearest neighbour (k-NN) algorithm [6]. Random forest (RF) is one of the widely used machine learning models for classification tasks that uses “wisdom of the crowd” to make the final prediction. RF is a good choice when it comes to the problem of high dimensional and imbalanced data [7, 8]. The accuracy is better than other machine learning models as it uses the mean or average of many decision trees for the final decision. Currently, it is being employed in many domains like health care, prediction for time series data and agriculture, etc. [9, 10].

In general, this study makes the following contributions:

- A methodology is designed to perform automatic rose classification using rose leaves. For this purpose, the image processing approach is followed. Two sets of features are tested for this task including histogram and texture features. Four subsets of features are evaluated through extensive experiments.
- The performance of Naive Bayes (NB), Generalized Linear Model (GLM), Deep Learning (DL) Multinomial Model, Decision Tree (DT), RF, Gradient Boosted Trees (GBT), and Support Vector Machine (SVM) is analyzed in detail. For experiments, a new dataset of rose leaves is collected.
- Ensemble classifiers are tested for the classification task using various combinations of selected machine learning models with four subsets of features to analyze the classification accuracy.
- This study especially focuses on the performance of RF which shows better results than other models for rose plant classification. Due to good results of RF, its performance is further improved by analysing the influence of various selection criteria such as Information Gain, Gini Index, etc.

The rest of the paper is organized as follows.  Section 2 discusses research papers from the literature which are closely related to the current study.  Section 3 gives an overview of the machine learning algorithms adopted for the current research, the description of the dataset used for the experiment, as well as, the proposed approach. Results are discussed in Section 4. In the end, the conclusion is given in Section 5.

## 2. Literature Review

Classification of plants carries multiple purposes such as to name plants, extract useful information, study features that impact yield of fruits/vegetables and quality, and predict their price. Some representative classification approaches are presented next.

### 2.1. Machine Learning Models

Machine learning offers reliable algorithms for predictability [11, 12]. For predicting prices of various varieties of fruits, they have been classified using a hybrid method based on texture, histogram and colour features [13]. The proposed algorithm FSCABC–FNN obtained 89.1% classification accuracy. Tomatoes have been graded for readiness using colour traits in [14]. Principal components analysis and SVM are used for feature extraction and linear discriminant for categorization. Results show 90.80% accuracy. Quality assessment and disease detection of sunflowers using texture and colour traits obtained from leaves has been studied using multi-class SVM, k-NN, Multinomial Logistic Regression, and NB in [15]. Another work suggests the importance of structural cues for flower identification [16]. The feature vector is built and input to the proposed method. The accuracy is increased from 76.9% to 82.6%. A performance comparison for classification of plants using computer vision is presented in a survey [17]. Plant organs, information on different features namely vein structure, colour, shape, margin, and texture are studied. Texture features in combination with leaf traits are found to be the best for identification.

The authors build a vision-based leaf identification system in [18]. The study uses different features including the shape, inner structure, colour, surface For this purpose. Similarly, [19] designs a mobile-based leaf identification system that first determines the leaf and non-leaf samples and then classifies the leaves. Curvature-based shape features are used in this regard. Experimental results show the efficiency and robustness of the proposed system. Rose plant classification is carried out in [6] that deploys k-NN based approach to this end. Using a different number of neighbours for k-NN, experiments are performed with histogram and texture features. The obtained accuracy for histogram and texture features are 65.00% and 45.50%, respectively. Similarly, [20] endeavours to classify eight types of flowers using scale-invariant feature transform (SIFT) features. SVM and RF are applied for the classification of the features from segmented images. Rather a short dataset containing 215 images is used for classification where high accuracy is achieved when flowers of dissimilar shapes are classified. The authors use pre-trained VGG16 architecture to rose flower disease classification in [21]. Early and late fusion techniques are applied combining VGG16 and SVM where the early fusion models show better results with 88.33% accuracy. The study [22] provides a comprehensive review of machine learning models that are recently adopted for species classification. The study especially covers the vision-based approaches applied for flower classification and discusses the famous pre-trained models.

An AI-based guava disease prediction system is presented in [23] that utilizes the high-quality images of guava leaves. The efficiency of several machine learning classifiers is evaluated like k-NN, complex tree, boosted tree, bagged tree, and SVM. Additionally, the use of histogram and textual features prove to show higher accuracy.

### 2.2. Use of Deep Learning Models

Predictability through deep learning promises improvement over machine learning algorithms, as demonstrated in various dynamic problem areas such as cloud computing [24]. In the context of this work, the quality and defects of the Jasmine flower have been identified with an 83% efficiency using texture, colour, and shape traits [25]. Plants have been identified using leaf features with images taken directly from plants [26]. The used method is based on a convolutional neural network (CNN) and features based on a deconvolutional network. It is found that shape features are inadequate for identification due to less discriminatory information contained in the leaves. On the contrary, venation structure and leaf shape features give better results. Similarly, species classified using deep learning is found a promising approach [27]. A non-scalable manual approach is proposed in which visual characteristics have been selected from flower images and generalized to predict new unknown flowers [28]. The proposed method proved to be more effective than traditional approaches. There have been efforts to understand roses in detail and to recognize their variety [29]. The work is based on Fourier Transformation that considers descriptor angles of roses to recognize their shapes like round, irregular round, or star. The obtained efficiency is higher than other contemporary methods. Similarly, a system of neural network-based classification has investigated blooming flowers [30]. A detailed analysis of different machine learning classifiers like NB, DT, simple k-Means, MLP, SVM, and RF using the WEKA tool is presented in [31]. The main objective is to find the best classification algorithm to enhance the accuracy of classification with reduced processing time. Many evaluation parameters are used for analysing results such as mean absolute error, root means squared error, TP-rate, TN-rate, FP-rate, FN-rate, precision, and recall. Results indicate NB is the best choice for improving traditional classification problems. SVM gives the best average accuracy.

Plant classification using a CNN is performed in [32] which used the BJFU100 dataset containing 100 species of iris plant. Images are added to the dataset using a mobile device application to collect more images. The residual network is introduced which removes the vanishing gradient and degradation problems. The proposed network is 26 layers in-depth and allows the input flow to deeper layers without losing information. The parameters of RestNet26 are well trained that they can learn the discriminative features and avoid under fitting. The proposed approach can achieve an accuracy of 91.78% which is better than the existing RestNet with 18, 34, and 50 layers. Another deep learning approach called a Fully Convolutional Network (FCN) is proposed in [33] for plant classification. It performs automatic segmentation of flowers from the background. It used the VGG-16 model for initialization. FCN has several convolutional layers and 3 deconvolutional layers. FCN is trained until the validation accuracy starts decreasing and training is restarted from the last learned model. The objective is to let the model learn local features in the first two blocks. By this process they collected the segmented flower images and kept only those that had high discriminative region, other images are discarded. A CNN is proposed to be trained on FCN. Evaluation metrics are proposed for measuring the accuracies of the segmentation, detection, and classification methods. Results show the accuracy of 99.0%, 98.5%, and 97.1% on Zou-Nagy, Oxford 17, and Oxford 102, respectively.

Along the same lines, [34] presents the use of multiple deep learning models and combines auto encoders and CNN for plant leave classification. The auto encoder and CNN are used for feature extraction which is later used to train an SVM for classification which yields better results than traditional machine learning models. The authors utilize low-quality images in [35] with deep learning models to improve the performance for plant disease prediction. The study utilizes Chebyshev orthogonal functions and probability distribution functions regarding the colour histograms. Experiments performed using the MobileNetV2 show better performance over traditional methods. Similarly, a mask residual CNN (RCNN) based approach is presented in [36] recognizing to detect diseases from apple leaves. Experiments using the Plant Village dataset yield a 96.6% accuracy using the ensemble subspace discriminant analysis. In a similar fashion, a residual NN (RNN) is used by authors in [37] for detecting cassava mosaic disease. A modified deep RNN is designed for disease detection with a balanced dataset using block processing. With a balanced dataset high accuracy is reported with deep RNN showing 9.25% better performance than a traditional CNN.

### 2.3. Use of Selective Features for Classification

A flower classification technique is introduced in [38] which uses selective discriminative features for 103 class datasets. Images are downloaded from the web which varies in scale, resolution, clutter, lighting, quality, etc. An automatic segmentation scheme introduced by Nilsback and Zisserman is used. Colour, histogram of gradient (HOG) features are used using SIFT for the foreground region. SVM is used as a classifier where each kernel represents each feature. Classification results are much better with combined features within the kernel framework, which improves efficiency. Study [39] described different perspectives of image acquisition and its impact on classification accuracy. Three image factors are considered: perspectives, illumination, and background. CNN is used for feature extraction and SVM for classification. Total 27 datasets are formed using nine image types (backlight on/off, plain background/natural background, top view, and back view of the leaf) and three pre-processing strategies are used pre-processed, cropped, and segmented. The highest accuracy of 91% on cropped backlight images and 55% lowest accuracy is achieved on non-pre-processed images. It is found that cropping is more effective than segmenting, backside images do not contribute to achieving higher accuracy but need more human efforts in image acquisition. The non-destructive way is to take topside images and crop them from leave boundaries of herbaceous leaves. If the destructive way is permissible plucking the leaf using backlight yields higher accuracy. Spatio-temporal features have also been utilized with deep learning models for prediction and classification as in [40] for crow flows prediction. Similarly, the Spatio-temporal features are used with hybrid deep learning models in [41]. An attention-based network is designed in [42] that makes use of Spatio-temporal features for traffic flow prediction.

The authors developed an image capturing scheme in [43] for obtaining the best perspectives that contribute to the classification accuracy of flowering plants. The images of a single plant are taken considering five different perspectives: entire plant, flower frontal, flower lateral, leaf top, and leaf back. A large dataset comprising 101 species of plant families is assembled. Images are taken during the flowering season. A CNN is trained on the collected dataset shows that CNNs can learn the discriminative features directly from raw pixels. Transfer learning is used for training while the performance is evaluated using a simple sum rule that combines the scores of different perspectives. An accuracy of 77.4% is achieved for the entire plant, 88.2% for flower frontal, and the best results are achieved by fusing all five perspectives giving an accuracy of 97.1%. It is concluded that the species that are difficult to recognize even by humans can be recognized by multi-organ identification. Because of the lack of a universal perspective for all species, different organ views of the plant are beneficial for identifying the important perspectives of plants.

## 3. Methodology

In this section, we discuss the proposed methodology. The steps followed in the proposed methodology are shown in Figure 1 and briefly described in the preceding sections.

### 3.1. Data Collection

Machine learning algorithms learn on the available data or evidence. Mistakes in data collection are easily propagated to the training phase and affect the performance of classifiers. Thus, we have collected data carefully using a 23MP camera capturing orange, red, pink, and white rose leaves (please see Figure 2). Images are taken in a controlled environment keeping the light condition the same for all images. Each image comes from a different plant. The images are captured in a controlled environment where the lighting conditions are almost similar for all the captures. The dataset consists of 10 classes. The resolution of the captured image is 1080 × 1920 pixels. The data is split into 0.6 to 0.4 ratios for training and testing, respectively.

### 3.2. Data PreProcessing

We convert colour images to grey level images and mark two regions of interest (ROIs) on each of them using the CVIP tool [44]. Thus, dataset of size 200 is formed. Conversion into grey level aims at reducing the unnecessary information from the images and computational processing. Pre-processing allows feature enhancement and should be carried out carefully to avoid losing vital information that can lead to wrong identification.

### 3.3. Feature Extraction

Feature selection has a direct impact on the classification process. Feature space can easily grow enormously, hence extracting a minimal set of features is desirable though it is computationally intensive. Too much extraction of features may easily compromise generalization of results. Figures 3 and 4 show the examples of natural and artificial textures.

Table 1 shows the histogram and texture features used in this study. Each feature is defined next.

#### 3.3.1. Mean

Histogram mean describes the average level of intensity of the image or texture being examined [45]. Mathematically it is given as,

(1) $$\begin{array}{c} \mu =\sum_{i=0\;}^{G-1}i\times p\left(i\right), \end{array}$$

where *p(i)* is the fraction of samples in class *i* and *G* is the number of grey levels used [6].

#### 3.3.2. Skew

Skewness provides the data with distribution, whether or not the resulting distribution is symmetric, positively skewed, or negatively skewed [31]. It is given as [6],

(2) $$\begin{array}{c} \mu_{3}=\sigma^{-3}\sum_{i=0\;}^{G-1}{\left(i-\mu \right)}^{3}\times p\left(i\right). \end{array}$$

#### 3.3.3. Energy

Energy feature measures the contrast between a pixel and its surrounding pixels [32]. It gives a large value if the image is homogeneous. Homogeneous means there are a large number of pixels that have similar intensity values. If this feature gives a positive 1, it means the image is constant. It is given as,

(3) $$\begin{array}{c} \sum_{i=0\;}^{G-1}\sum_{j=0}^{G-1\;}{\left[p\left(i,j\right)\right]}^{2}, \end{array}$$

where *i, j* are the spatial coordinates of the function *p*(*i*, *j*) [6].

#### 3.3.4. Entropy

It varies inversely with the energy, while it is defined as the number of bits needed to code the data [46]. It is given as,

(4) $$\begin{array}{c} \sum_{i}\sum_{j}p\left(i,j\right)\times \;\log\left(p\left(i,j\right)\right), \end{array}$$

where *i* and *j* are the fractions of examples in class *i* and *j*, respectively [6].

#### 3.3.5. Inertia

Inertia is an image moment and shows a weighted average in terms of intensity of image pixels. It is calculated using

(5) $$\begin{array}{c} \sum_{i=0}^{G-1}\sum_{j=0}^{G-1\;}{\left(i-j\right)}^{2}\times p\left(i,j\right), \end{array}$$

where *i, j* are the spatial coordinates of the function *p(i, j)* [6].

#### 3.3.6. Correlation

It is the relationship between two values. The coefficient of correlation lies between 1 and −1. A value near 1 means there is a positive correlation between nearest pixel values, while a value closer to -1 means there is a negative correlation between them [32, 46]. It is given as

(6) $$\begin{array}{c} \sum_{i=0}^{G-1}\sum_{j=0}^{G-1\;}\frac{i\times j\times p\left(i,j\right)-\mu_{x}\times \mu_{y}}{\sigma_{x}\times \sigma_{y}}, \end{array}$$

where *μ*_*x*_ and *μ*_*y*_ are the means and *σ*_*x*_ and *σ*_*y*_ are the standard deviations of *p*_*x*_ and *p*_*y*_, the partial probability functions [6].

#### 3.3.7. Inverse Difference

It is the local homogeneity that is high when the local grey level is uniform [46, 47]. It is given as

(7) $$\begin{array}{c} \sum_{i=0}^{G-1}\sum_{j=0}^{G-1\;}\frac{p\left(i,j\right)}{1+{\left(i-j\right)}^{2}\;}, \end{array}$$

where *p(i, j)* is the probability that a pixel with value *i* will be found adjacent to a pixel of value *j* [6].

Selection of histogram and texture features is based on their success rate in similar classification problems [48–51]. The contribution of histogram due to its brightness and contrast aspects is proven [30]. For classification through leaves texture feature has a vital role. Texture not only considers leaf venation structure but also gives the directional characteristics of pixels selected from the leaf. It is independent of leaf colours and shape. Texture analysis is made from a group of pixels. It is considered more dominant a feature than the shape feature [5, 17].

CVIP is a famous library used for simple to complex image processing tasks like image reading, transforming, and region of interest (ROI) capturing [52]. It also provides automated tools to control the quality of images and image enhancement. It is used with a graphical user interface (GUI) based software tools like LabView where numerical and statistical analysis can also be performed.

### 3.4. Deep Learning Models

In addition to machine learning models, this study implements deep learning models for rose plant classification.

#### 3.4.1. Convolutional Neural Network

CNN is a widely used deep learning model for image processing tasks [1]. Good results can be obtained by CNN as it can efficiently handle data complexity and pre-processing. It includes a convolutional layer to learn complex features from the input data while max-pooling is used as the pooling layer in this study. The convolution layer is used with rectified linear unit (ReLU) activation while the kernel size is 3 × 3. Max-pooling is used with 2 × 2. It is followed by a flatten layer and 0.2 dropout layer to reduce the probability of model over fitting. A dense layer is used with 512 neurons.

#### 3.4.2. Long Short-Term Memory Network

This study also uses the LSTM model for rose plant classification. LSTM has four gates, each for a different task. LSTM has a feedback mechanism and produces good results for classification tasks [53]. LSTM is used for an embedding layer with dimensions of 5000 and 100. It is followed by a dropout layer with a 0.5 dropout rate. Then an LSTM layer is added with 100 units. In the end, a dense layer is added with a “softmax” activation layer to get the output for the desired number of classes.

#### 3.4.3. RestNet

The RestNet also called residual network is a pre-trained model and is among the commonly used pre-trained models for tasks related to image processing. RestNet aims at providing high accuracy for complex image processing tasks [54]. It has different layers where each layer has a different structure with respect to convolutional size and filters. Possessing a deep structure, RestNet can learn better by going deeper during the training phase and ultimately provides better results than traditional deep learning models [55].

## 4. Results and Discussion

We used CVIP tool to extract features and RapidMiner [56] for classification. Small result subsets of texture and histogram related features are listed in Tables 2 and 3, respectively. The rest of the results are not listed for brevity.

### 4.1. Formation of Feature Sets

In this work, results were obtained by using seven different classifiers as described above. We made four feature sets by using the auto model of the RapidMiner tool. These feature sets are made by selecting the features from the set of Histogram and Texture features which are extracted from the images of rose leaves. Results obtained by all classifiers on these feature sets are different for a different set of features. Different sets of features are described below.

#### 4.1.1. Feature Set 1

All extracted features of histogram and texture are used to make feature set 1 (FS1). Histogram mean, histogram standard deviation, histogram energy, histogram skew, histogram entropy, texture energy average, texture energy range, inertia average, inertia range, correlation average, correlation range, inverse difference range, inverse difference average, and texture entropy average.

#### 4.1.2. Feature Set 2

Features having a high correlation with the label column are selected from both histogram and texture features to make feature set 2 (FS2). Histogram mean, histogram standard deviation, histogram energy, histogram entropy, texture energy average, texture energy range, inertia average, inertia range, inverse difference range, and texture entropy average.

#### 4.1.3. Feature Set 3

Feature set 3 (FS3) contains only histogram features with a high correlation to the label column. Histogram mean, histogram standard deviation, histogram energy, and histogram entropy.

#### 4.1.4. Feature Set 4

Set of all texture features with high correlation to labels are used to make feature set 4 (FS4). Texture energy average, texture energy range, inertia average, inertia range, inverse difference range, and texture entropy average.

### 4.2. Error Metrics

To correctly evaluate the performance of classifiers confusion matrices are used which have four different values. True positive (TP) show the number of those instances that are classified correctly, true negative (TN) represent instances that are true but classified incorrectly, false negative (FN) represent those instances that are false and classified as false while false positive (FP) represents the number of instances that are false but classified as true. Based on these values precision and recall can be evaluated [13].

Recall: This term represents the probability that how many positive classes are recalled by our classifier. The term is defined by
  (8) $$\begin{array}{c} \text{Recall}=\frac{\text{TP}}{\text{TP}+\text{FN}}. \end{array}$$
Precision: This term represents the probability that how many true positives were found by our classifier. The term is defined by
  (9) $$\begin{array}{c} \text{Precision}=\frac{\text{TP}}{\text{TP}+\text{FP}}. \end{array}$$

In the end, the classification error is used which represents the percentage of incorrect class predictions.

### 4.3. k-Nearest Neighbour

In our previous work we used CVIP for k-NN to obtain results on histogram and texture features, the obtained accuracy is 65% and 45.50%, respectively [6]. We formed two feature sets including histogram features and texture features.  Figure 5 shows the result of k-NN on different values of *k*.

### 4.4. Parameter Settings of Machine Learning Models

We tuned some general parameter settings of machine learning models in RapidMiner and the rest of the parameters are used by their default values. The split operator in the process model makes partitions of data as training set and testing set. It takes 60% examples for training and 40% for testing. Another parameter is sampling types which are automatic, linear, shuffled and stratified. For nominal data types, we used stratified sampling.

The parameter settings of NB have the Laplace correction parameter which avoids the conditional probability set to zero and also avoids misleading results. It is a kind of Boolean operator with a default value that is true.

GLM has a few parameter settings: family, solver, the maximum number of threads, and regularization. The family parameter has different types including Gaussian, Binomial, Poisson, Gamma, Multinomial, Tweedie, and Auto. Gaussian is used for numeric data (real or integer), Binomial for binomial data, Multinomial for polynomial data more than two classes, Poisson is used for numeric and non-negative data, Gamma is applied for continuous, numeric, and positive data, Tweedie is used for numeric, continuous and non-negative and Auto option selects multinomial for polynomial, binomial for binomial and Gaussian for numeric data. Solver parameter includes IRLSM, L_BFGS, Coordinate_Descent_Naive and Coordinate_Descent. IRLSM is useful for the problems which have a small predictor size, L_BFGS better works on the dataset with many columns, Coordinate_Descent_Naive and Coordinate_Descent are the updated versions of IRLSM. The maximum number of threads is used to make the model reproducible and its default value is 4. Regularization uses the lambda and alpha parameters for controlling the regularization and distribution respectively. Standardize is used for numeric columns to have zero mean and unit variance. A complete list of all parameters used for the machine learning models is provided in Table 4.

Parameters for DL multinomial model are activation function, hidden layer sizes, epochs, adaptive learning and standardization. The activation function is used by neurons in the hidden layers to normalize the output. The activation function is of types Tanh, Rectifier, Maxout and ExpRectifier. The hidden layer size parameter is used to change the size of hidden layers. Epochs are used for iterating the dataset. Adaptive learning is used to avoid the slow convergence by combining learning rate and momentum training. For this purpose, it uses epsilon and rho. Standardize is used for regularization, it has different parameters; L1, L2, max w2, loss function, and distribution function. The loss function is of types Automatic, Quadratic, CrossEntropy, Huber, Absolute, and Quantile. The distribution parameter has sub-parameters of type Auto, Bernoulli, Gaussian, Poisson, Gamma, Tweedie, Quantile, and Laplace.

DT parameters include criterion, maximal depth, pruning, and pre-pruning. Criterion includes Gain Ratio Information Gain, Gini Index, Accuracy, and Least Square. Maximal depth is used for varying the size of the tree according to example set. If the pruning parameter is checked it will replace some branches with leaves according to the confidence parameter and pre-pruning specifies the stopping criteria for the generation of the tree. Random Forest parameters are the same as DT except for the additional parameter number of trees. GBT parameters are the number of trees, maximum number of threads, maximal depth, learning rate, sample rate, and distribution. The distribution parameter has the same types that were defined for Deep Learning.

SVM parameters include SVM type, kernel type, gamma, C, cache size, epsilon, shrinking, and confidence with multi-class. SVM type is used to select the type of SVM which are C_SVC, nu_SVC, one_class, epsilon_SVR, and nu_SVR, first two types are used for classification tasks, epsilon-SVR and nu-SVR are used for regression, and distribution estimation one-class SVM is used. Kernel type parameter includes linear, poly, RBF, sigmoid, and pre-computed. RBF kernel is the default type; it maps the samples into high dimensional space using a nonlinear function. Gamma is used with poly, sigmoid, and RBF kernels and play important role in changing the accuracy of the model. C specifies the cost parameter and it is used with SVM types C_SVC, epsilon_SVR, and nu_SVR. Epsilon is used for termination criteria.

Tables 5–8 show precision, recall, classification error and accuracy of all classifiers on feature sets FS1, FS2, FS3 and FS4.

In Figure 6 it is shown that precision, recall, and accuracy of NB and DT are lower than other classifiers. The higher the accuracy, the lower will be the classification error. SVM obtained the highest accuracy of 72% on FS1 as compared to other classifiers.

Accuracy depends on both values of precision and recall. Figure 7 shows the comparison of all classifiers. Here RF, DL, and SVM achieved equal accuracies on FS2. DT showed improvement on this data set by obtaining an accuracy of 60% which was 48% for FS1.

Classification results by all classifiers are depicted in Table 7 on FS3. This feature set only contains histogram features that have a high correlation with the labeled column. NB showed improvement on FS3 compared to FS1, FS2, and FS4.  Figure 8 shows that the precision, recall, and accuracy of all classifiers are the same on FS3.

Classification results on FS4 are less than other feature sets. All classifiers achieved low accuracy on FS4 because this feature set only contains the texture features with a high correlation to the label column. Texture features alone are not good features for classification tasks when there is a small dataset because it works on patterns.

Precision, recall, classification, and accuracy on FS4 are shown in Figure 9. It is shown that the accuracy lies between 34% and 45% which is very low than other feature sets.

Table 9 shows the accuracy of all classifiers on four feature sets. SVM gave the highest accuracy of 72% on FS1 and lowest accuracy of 34% on FS4.

### 4.5. Ensemble Learning

Ensemble learning is the technique of integrating multiple learners to solve the same problem. It builds multiple sets of hypotheses from training data and uses them together. The generalization ability of the ensemble is greater than the individual learners. It provides a more robust solution where the dataset does not contain equal distribution. The first step is to generate base learners either in a parallel manner or sequential and the second step is to combine all base learners for producing multiple combinations, majority voting and weighted averaging are the popular combination schemes for classification and regression respectively. The accuracy of the ensemble methods can be estimated by cross-validation, hold-out test, etc. For the construction of a useful ensemble method, it needs to consider multiple measures, e.g., subsampling the training examples, manipulating the features, manipulating the output and random integration of algorithms. Bagging, boosting, and voting are the common techniques for combining the algorithms [57].

In our study, we used the voting method to combine the algorithms. First, we carried out experiments for each algorithm, and then their results were combined for each instance of the test data. The instance with the highest votes of a class label has given that label. We used NB, GLM, DT, DL, RF, GBT, and SVM for producing ensemble results. We made eleven combination sets by integrating algorithms. The first set contains all seven algorithms, the second set five algorithms (GLM, DL, RF, GBT and SVM) that achieved higher accuracies and the third set nine random combinations of three algorithms from the second set. Results of these ensemble algorithms on our four feature sets are given in Table 10.

The results shown in Table 10 are obtained by integrating the output of each algorithm with the output of other algorithms of each instance by voting mechanism. The accuracy obtained by ensemble algorithms is better than individual algorithm accuracy, only SVM accuracy is higher than the ensemble algorithms accuracy.

### 4.6. Performance Optimization of Random Forest

We carried out performance optimization of RF results towards the improvement of accuracy. To this end, various combinations of the number of trees and the depth of trees are tested. The number of trees is varied from 2 to 102 with a difference of 10 and the depth of trees from 1 to 100 with the same difference. It is worth mentioning that Rapidminer uses Gain Ratio as an attribute selection criterion for RF as a general approach, though it does not explicitly disclose the value used for the Gain Ratio. We handle this situation concretely for our case by testing the impact of explicit values of the Gain Ratio. Additionally, we also tested two other attribute selection criteria, Information Gain and Gini Index.

Results obtained by optimized RF with Gain Ratio achieved higher accuracy than Information Gain and Gini Index. Results obtained by tuning the number of trees and depth of trees with Gini Index, Information Gain, and Gain Ratio as attribute selection criteria are given in Tables 11–23.

#### 4.6.1. Information Gain

Table 11 shows the optimized results of RF by varying the number of trees and depth of trees with selecting the Information Gain as an attribute selection criterion. There is no change in results by tuning the number of trees and depth of trees.

Table 12 shows no change in results with Information Gain also on FS2 by tuning the parameters of RF.

Results depicted in Tables 13 and 14 show that using Information Gain as attribute selection criterion with tuning the parameters of RF does not have any impact on accuracy. Results show consistent value by varying the number of trees and their depth. But accuracy for different feature sets is different.

#### 4.6.2. Gini Index

Tables 15–18 shows the results of RF by varying its parameters with Gini Index as attribute selection criterion. Results obtained by Gini Index are similar to results obtained by Information Gain by giving the single constant value with no difference in classification accuracy.

#### 4.6.3. Gain Ratio

Tables 19–22 show the accuracy achieved by varying the number of trees and its depth with Gain Ratio. Results obtained with the Gain Ratio are better than Information Gain and Gini Index. Gain Ratio gives the highest accuracy of 75.6% with 12 trees and 11 depth on FS1.

In Figure 10 it is shown that the maximum accuracy was achieved with 12 trees and 11 depth. After increasing the number of trees and depth from 12 to 11 respectively, accuracy is decreased instead of increasing. But this accuracy is greater by 13% than auto model results of RF on FS1.

Maximum accuracy obtained on FS2 is 78% with Gain Ratio. These results are greater than the results of the auto model of RapidMiner tool which was 69% on FS2. Results are given in Table 20.

Figure 11 shows the result of optimized RF on FS2. The highest accuracy is achieved with 22 trees and 11 depth. Accuracy is decreasing beyond 32 trees and 11 depth.

Results on FS3 are shown in Table 21. The maximum accuracy achieved on FS3 is 70.73%. Results of optimized RF are 2% greater than the auto model of RF on FS3. The result of optimized RF on FS3 is shown in Figure 12.

Table 22 shows the results on FS4. Accuracy on FS4 is 51.7% which is less than other feature sets but greater than auto model accuracy. The result of optimized RF on FS4 is shown in Figure 13. Comparison using Information Gain, Gini Index, and Gain Ratio as an attribute selection criterion is depicted in Table 23 and it is shown that Gain Ratio obtained higher accuracy than others.

### 4.7. Performance of Deep Learning Models

Besides using machine learning models and optimizing the performance of RF, this study conducted experiments using deep learning models. Table 24 shows the results of deep learning models, which indicate that the performance of deep learning models is poor as compared to results obtained with FS2 using RF classifier. Apparently, the small size of the data is not large enough for the deep learning models to learn the complex relationships. Similarly, for proper training, RestNet could not find a large feature set and its performance is lower than expected. Deep learning models are data-intensive and do not perform well when the data size is small [58].

### 4.8. Results Using k-Fold Cross-Validation

To confirm the performance of the used machine learning models and RF model especially, k-fold cross-validation is performed as well.  Table 25 shows the results of 10-fold cross-validation for all the models used in this study. Results show that RF provides the highest accuracy of 0.78 followed by LSTM for the rose plant classification task. RF performance is compared with FS2 where its accuracy is the highest of all models.

### 4.9. Results of T-Test

For corroborating the performance of RF over other models, the statistical *T*-test is performed with the following hypotheses:

- Null Hypothesis (H0): The performance of RF is not statistically significant over other approaches.
- Alternative Hypothesis (Ha): The performance of RF is statistically significant over other approaches.

Accepting the H0 indicates that the performance of RF and other models is similar with no substantial difference. On the other hand, rejecting the H0 and accepting the Ha confirms that the performance of other models and RF has substantial differences and RF shows superior performance to other models. For this study, the *T*-test rejects the H0 and accepts Ha as the value of *t* is 4.769 with a critical value equal to 0.491.

## 5. Conclusion

The current study aims to classify the rose plant leaves using NB, GLM, DL, DT, RF, GBT, and SVM; in essence, the performance of RF is extensively investigated. Several sets of experiments have been performed with histogram features and texture features. For analysing the efficacy of various combinations of these features, four feature sets are made concerning their correlation to the target class. Results indicate that SVM obtains the highest accuracy of 72% on FS1. The FS1 contains both texture and histogram features having a high correlation with the target class both features contribute to classification. Other classifiers show better performance when trained on FS2 and FS3. But the performance of all classifiers is poor on FS4 because it contains only texture features which indicate that using texture features alone is not useful for predicting true labels. A special emphasis is placed on ensemble models and various combinations of selected classifiers are used in this regard. The accuracy achieved by ensemble learning is higher than individual algorithms except for SVM. Owing to its better performance, RF is investigated in detail by varying the number of trees, its depth, and attribute selection criterion including Information Gain, Gini Index, and Gain ratio. This parameter tuning contributes to achieving better accuracy than using a model as the black box. The optimization of RF proves to show better results than the auto model. RF achieves the highest accuracy scores of 73.17% with Information Gain, 78.05% with Gini Index, and 78.0% with the Gain ratio for FS3, FS2, and FS2, respectively. The bias of Information Gain towards choosing the attributes with more information values leads to poor performance than that of Gain ratio and Gini Index. In addition, CNN, LSTM, and RestNet models are used for experiments, however, their performance is not better than the fine-tuned RF. Owing to the small size of the dataset, the performance of the deep learning models is not investigated extensively. We intend to enlarge the dataset size by collecting further images and utilizing the resampling techniques as well. We also plan to compare the performance analysis of other classification algorithms such as neural networks, SVM, and DT for rose classification problems. Also, it would be interesting to select features methodically.

## Figures and Tables

**Figure 1:** Steps followed in the proposed methodology. Starting with data collection, study follows data processing before feature extraction. In the end, classification is performed.

**Figure 2:** Leaves of different colored roses, (a) Orange rose, (b) Pink rose, (c) Red rose, and (d) White rose. The leave images are from the dataset collected for experiments in this study.

**Figure 3:** Examples of artificial textures.

**Figure 4:** Examples of natural textures.

**Figure 5:** Performance of k-NN on texture and histogram features.

**Figure 6:** Results of Machine Learning classifiers when trained using the FS1.

**Figure 7:** Results of Machine Learning classifiers when trained on FS2.

**Figure 8:** Results of Machine Learning classifiers when trained with FS3.

**Figure 9:** Results of Machine Learning classifiers when trained with FS4.

**Figure 10:** Impact of different number of trees and depth on accuracy of FS1 choosing Gain Ratio as attribute selection criteria.

**Figure 11:** Impact of different number of trees and depth on accuracy of FS2 choosing Gain Ratio as attribute selection criteria.

**Figure 12:** Impact of different number of trees and depth on accuracy of FS3 choosing Gain Ratio as attribute selection criteria.

**Figure 13:** Impact of different no. of trees and depth on accuracy of FS4 choosing Gain Ratio as attribute selection criteria.

**Table 1:** The list of features used for different classifier.

Histogram features	Texture features
Mean	Energy
Standard deviation	Inertia
Skew	Correlation
Energy	Inverse difference
Entropy	Entropy

**Table 2:** Few sample results of histogram features.

Labels	ROI	Mean	Standard deviation	Skew	Energy	Entropy
Orange	1	29.488	3.531	0.464	0.084	3.790
	2	28.568	4.100	0.222	0.068	4.023
	3	32.147	7.296	0.160	0.040	4.837

Red	1	31.249	2.079	0.053	0.140	3.075
	2	22.422	0.999	0.341	0.295	2.013
	3	28.989	2.355	0.246	0.121	3.237

White	1	38.696	3.034	1.587	0.133	3.334
	2	54.209	2.494	0.262	0.116	3.347
	3	64.674	3.340	0.397	0.086	3.757

Pink	1	78.337	2.419	0.444	0.121	3.271
	2	73.467	2.579	0.903	0.123	3.288
	3	63.028	2.686	0.273	0.106	3.451

**Table 3:** Few sample results of texture features.

Labels	ROI	Energy	Inertia	Correlation	Inverse difference	Entropy
Orange	1	0.0103	4.295	0.248	0.532	0.543
	2	0.002	14.519	0.306	0.434	0.400
	3	0.001	8.940	0.241	0.493	0.244

Red	1	0.041	0.894	0.238	0.432	0.351
	2	0.009	2.934	0.268	0.509	0.271
	3	0.013	1.657	0.234	0.516	0.299

White	1	0.002	7.570	0.223	0.499	0.266
	2	0.001	16.115	0.248	0.425	0.175
	3	0.002	7.304	0.211	0.496	0.307

Pink	1	0.001	14.272	0.230	0.429	0.115
	2	0.001	8.712	0.364	0.468	0.124
	3	0.001	35.020	0.491	0.340	0.317

**Table 4:** The parameters used for the machine learning models.

Machine learning models	Tuning parameters	Values used
NB	Laplace correction	Yes

GLM	**Family (**Gaussian, binomial, Poisson, gamma, tweedie, auto)	Auto
	**Solver** (IRLSM, L_BFGS, Coordinate_Descent, C_D_Naive)	Auto
	No. of threads	1
	Regularization	Lambda, alpha

DL	**Activation function** (tanh, rectifier, maxout, ExpRectifier)	Rectifier
	Hidden layer size	50
	Epochs	10
	Adaptive learning	Epsilon, rho
	Standardize	Loss function, distribution function

DT	**Criteria** (Gain_Ratio, Information_Gain, gini index, accuracy, Least_Square)	Gain_Ratio
	Maximal depth	7
	Pruning	Yes
	Prepruning	Yes

RF	No. of trees	100
	Maximal depth	7
	Criterion	Gain_Ratio

GBT	No. of trees	60
	No. of threads	1
	Maximal depth	4
	Learning rate	0.1
	Sample rate	1.0
	Distribution	Auto

SVM	**SVM type** (C_SVC, nu_SVC, one_class, epsilon_SVR, nu_SVR)	Rectifier
	Kernel type	rbf
	C	1000.0
	Cache size	80
	Epsilon	0.001

**Table 5:** Precision, recall, and classification error on FS1.

Classifiers	Precision (%)	Recall (%)	Classification Error (%)	Accuracy (%)
NB	54	40	60	40
GLM	67	64	35	65
DL	71	68	31	69
DT	49	46	52	48
RF	60	60	38	62
GBT	66	67	32	68
SVM	71	71	28	72

**Table 6:** Precision, recall, and classification error on FS2.

Classifiers	Precision (%)	Recall (%)	Classification error (%)	Accuracy (%)
NB	49	41	58	42
GLM	60	59	40	60
DL	74	69	31	69
DT	62	59	40	60
RF	68	67	31	69
GBT	62	62	36	64
SVM	67	67	32	68

**Table 7:** Precision, recall, and classification error on FS3.

Classifiers	Precision (%)	Recall (%)	Classification error (%)	Accuracy (%)
NB	63	45	55	45
GLM	59	64	35	65
DL	75	66	34	66
DT	64	55	44	56
RF	69	67	32	68
GBT	70	68	31	69
SVM	70	64	34	66

**Table 8:** Precision, recall, and classification error on FS4.

Classifiers	Precision (%)	Recall (%)	Classification error (%)	Accuracy (%)
NB	35	38	60	40
GLM	45	40	58	42
DL	38	44	55	45
DT	28	40	59	41
RF	34	41	57	43
GBT	38	43	55	45
SVM	35	34	66	34

**Table 9:** Summary of classifiers accuracy (%) using different feature sets.

Feature sets	NB	GLM	DL	DT	RF	GBT	SVM
FS1	40	60	69	48	62	64	72
FS2	42	65	69	60	69	68	68
FS3	45	65	66	56	68	69	66
FS4	40	42	45	41	43	45	34

**Table 10:** Summary of ensemble classifiers accuracy (%) on different feature set.

Ensemble models	Accuracy (%)			
	FS1	FS2	FS3	FS4
NB + GLM + DT + DL + RF + GBT + SVM	66	60	63	39
GLM + DL + RF + GBT + SVM	70	67	67	35
GLM + DL + RF	65	65	66	43
GLM + DL + GBT	62	60	68	45
GLM + DL + SVM	65	65	65	40
GLM + RF + GBT	66	66	68	40
GLM + RF + SVM	66	67	67	36
GLM + GBT + SVM	68	63	67	35
DL + RF + GBT	66	67	67	41
DL + RF + SVM	67	69	66	39
RF + GBT + SVM	67	65	66	39

**Table 11:** Accuracy (%) results obtained by Information Gain on FS1.

No. of trees	Depth of trees					
	1	21	41	61	81	100
2	68.29	68.29	68.29	68.29	68.29	68.29
22	68.29	68.29	68.29	68.29	68.29	68.29
42	68.29	68.29	68.29	68.29	68.29	68.29
62	68.29	68.29	68.29	68.29	68.29	68.29
82	68.29	68.29	68.29	68.29	68.29	68.29
102	68.29	68.29	68.29	68.29	68.29	68.29

**Table 12:** Accuracy (%) results obtained by Information Gain on FS2.

No. of trees	Depth of trees					
	1	21	41	61	81	100
2	70.73	70.73	70.73	70.73	70.73	70.73
22	70.73	70.73	70.73	70.73	70.73	70.73
42	70.73	70.73	70.73	70.73	70.73	70.73
62	70.73	70.73	70.73	70.73	70.73	70.73
82	70.73	70.73	70.73	70.73	70.73	70.73
102	70.73	70.73	70.73	70.73	70.73	70.73

**Table 13:** Accuracy (%) results obtained by Information Gain on FS3.

No. of trees	Depth of trees					
	1	21	41	61	81	100
2	73.17	73.17	73.17	73.17	73.17	73.17
22	73.17	73.17	73.17	73.17	73.17	73.17
42	73.17	73.17	73.17	73.17	73.17	73.17
62	73.17	73.17	73.17	73.17	73.17	73.17
82	73.17	73.17	73.17	73.17	73.17	73.17
102	73.17	73.17	73.17	73.17	73.17	73.17

**Table 14:** Accuracy (%) results obtained by Information Gain on FS4.

No. of trees	Depth of trees					
	1	21	41	61	81	100
2	46.34	46.34	46.34	46.34	46.34	46.34
22	46.34	46.34	46.34	46.34	46.34	46.34
42	46.34	46.34	46.34	46.34	46.34	46.34
62	46.34	46.34	46.34	46.34	46.34	46.34
82	46.34	46.34	46.34	46.34	46.34	46.34
102	46.34	46.34	46.34	46.34	46.34	46.34

**Table 15:** Accuracy (%) results obtained by Gini Index on FS1.

No. of trees	Depth of trees					
	1	21	41	61	81	100
2	68.29	68.29	68.29	68.29	68.29	68.29
22	68.29	68.29	68.29	68.29	68.29	68.29
42	68.29	68.29	68.29	68.29	68.29	68.29
62	68.29	68.29	68.29	68.29	68.29	68.29
82	68.29	68.29	68.29	68.29	68.29	68.29
102	68.29	68.29	68.29	68.29	68.29	68.29

**Table 16:** Accuracy (%) results obtained by Gini Index on FS2.

No. of trees	Depth of trees					
	1	21	41	61	81	100
2	78.05	78.05	78.05	78.05	78.05	78.05
22	78.05	78.05	78.05	78.05	78.05	78.05
42	78.05	78.05	78.05	78.05	78.05	78.05
62	78.05	78.05	78.05	78.05	78.05	78.05
82	78.05	78.05	78.05	78.05	78.05	78.05
102	78.05	78.05	78.05	78.05	78.05	78.05

**Table 17:** Accuracy (%) results obtained by Gini Index on FS3.

No. of trees	Depth of trees					
	1	21	41	61	81	100
2	73.17	73.17	73.17	73.17	73.17	73.17
22	73.17	73.17	73.17	73.17	73.17	73.17
42	73.17	73.17	73.17	73.17	73.17	73.17
62	73.17	73.17	73.17	73.17	73.17	73.17
82	73.17	73.17	73.17	73.17	73.17	73.17
102	73.17	73.17	73.17	73.17	73.17	73.17

**Table 18:** Accuracy (%) results obtained by Gini Index on FS4.

No. of trees	Depth of trees					
	1	21	41	61	81	100
2	46.34	46.34	46.34	46.34	46.34	46.34
22	46.34	46.34	46.34	46.34	46.34	46.34
42	46.34	46.34	46.34	46.34	46.34	46.34
62	46.34	46.34	46.34	46.34	46.34	46.34
82	46.34	46.34	46.34	46.34	46.34	46.34
102	46.34	46.34	46.34	46.34	46.34	46.34

**Table 19:** Accuracy (%) results obtained by Gain Ratio on FS1.

No. of trees	Depth of trees					
	1	11	21	31	41	51
2	24.4	63.4	56.1	56.1	56.1	56.1
12	24.4	75.6	68.3	68.3	68.3	68.3
22	26.8	75.6	73.2	73.2	73.2	73.2
32	26.8	75.6	73.2	70.7	70.7	70.7
42	26.8	75.6	73.2	70.7	70.7	70.7
52	26.8	75.6	73.2	70.7	70.7	70.7

**Table 20:** Accuracy (%) results obtained by Gain Ratio on FS2.

No. of trees	Depth of trees					
	1	11	21	31	41	51
2	24.4	68.3	68.3	68.3	68.3	68.3
12	24.4	75.6	68.3	68.3	68.3	68.3
22	26.8	78	70.7	70.7	70.7	70.7
32	26.8	78	70.7	68.3	68.3	68.3
42	26.8	73.2	73.2	73.2	73.2	73.2
52	26.8	73.2	70.7	73.2	73.2	73.2

**Table 21:** Accuracy (%) results obtained by Gain Ratio on FS3.

No. of trees	Depth of trees					
	1	11	21	31	41	51
2	24.4	58.5	65.9	65.9	65.9	65.9
12	24.4	68.3	65.9	68.3	68.3	68.3
22	26.8	70.7	65.9	65.9	65.9	65.9
32	26.8	68.3	68.3	68.3	68.3	68.3
42	26.8	70.73	70.73	70.73	70.73	70.73
52	26.8	70.73	70.73	70.73	70.73	70.73

**Table 22:** Accuracy (%) results obtained by Gain Ratio on FS4.

No. of trees	Depth of trees					
	1	11	21	31	41	51
2	24.4	41.5	46.3	48.8	48.8	48.8
12	24.4	51.2	41.5	48.8	48.8	48.8
22	26.8	51.2	43.9	48.8	48.8	48.8
32	26.8	53.7	36.6	41.5	41.5	41.5
42	26.8	53.7	36.6	41.5	41.5	41.5
52	26.8	53.7	36.6	41.5	41.5	41.5

**Table 23:** Best results obtained by Gain ratio, Information gain and Gini Index (%) using different feature sets.

Feature sets	Gain ratio (%)	Information gain (%)	Gini index (%)
1	75.60	68.29	68.29
2	78	70.73	78.05
3	75.61	73.17	73.17
4	53.70	46.34	46.34

**Table 24:** Performance evaluation of deep learning models.

Model	Precision (%)	Recall (%)	F1 (%)	Accuracy (%)
CNN	0.72	0.72	0.70	0.72
LSTM	0.77	0.76	0.76	0.77
RestNet	0.74	0.72	0.73	0.74

**Table 25:** Results of 10-fold cross-validation.

Fold	NB	GLM	DT	RF	GBT	SVM
1st-fold	0.512	0.618	0.492	0.791	0.662	0.712
2nd-fold	0.522	0.671	0.487	0.780	0.638	0.722
3rd-fold	0.499	0.690	0.490	0.793	0.694	0.749
4th-fold	0.506	0.637	0.499	0.787	0.662	0.726
5th-fold	0.521	0.629	0.498	0.773	0.624	0.698
6th-fold	0.510	0.626	0.491	0.790	0.688	0.688
7th-fold	0.487	0.617	0.487	0.789	0.680	0.713
8th-fold	0.519	0.694	0.490	0.791	0.611	0.708
9th-fold	0.496	0.634	0.489	0.769	0.637	0.721
10th-fold	0.509	0.645	0.488	0.790	0.626	0.717
Average	0.508	0.646	0.491	0.785	0.652	0.715

## Data Availability

All data generated or analyzed during this study are included in this published article.
